# Problems and Countermeasures of China's Greenway Economic Development from the Perspective of Computer Internet

**DOI:** 10.1155/2022/6286833

**Published:** 2022-08-27

**Authors:** Shuping Zhang

**Affiliations:** Hotel Management Major, Department of Tourism and Foreign Languages, Ma'anshan Teacher's College, Ma'anshan, Anhui 243041, China

## Abstract

Given the advantages of urban greenways (UGCs) to urban populations' health and well-being, the growing usage of UGCs has gotten a lot of attention. However, most studies on UGCs have been undertaken in Western nations, but the understanding of greenway usage in underdeveloped countries is scarce. China's current environmental change in urban enhancement has been emphasized by a rush of urban green projects. The greenway is a kind of green infrastructure that has lately been the focus of many municipal governments. The federal government's new, ecologically friendly approach to urbanization is the subject of this article, which offers a preliminary assessment of the role played by greenways in that strategy. UGCs are green landscape routes designed for walkers and bicycles in cities, according to landscape design. A growing number of regions and cities in China are participating in the development of UGC, with some projects meeting their goals on an annual basis. UGCs are being built in China; however, a number of challenges exist, including a lack of legal basis, the public's incorrect understanding of UGCs, and insufficient scientific investigation. According to research on UGC construction and analysis of the peculiarities of various urban developments, the article highlighted current challenges in China's UGC construction and provided corresponding remedies in order to enhance China's UGC construction. In this survey, we performed statistical analysis using the chi-square test as well as the ANOVA test.

## 1. Introduction

China's economy has grown rapidly during the last few decades. By 2017, China's GDP had grown from 149.6 billion to 12.25 trillion USD, making it one of the world's wealthiest nations, with an additional 800 million people gaining access to better living conditions [1]. Increasing levels of environmental degradation, energy utilization, and industrial productivity have been associated with this growth [2]. Environmental deterioration, biodiversity loss, and soil erosion are all consequences of rapid economic growth.  Figure 1 illustrates the effect of environmental degradation by minimizing the environmental expenses of the nation. China's central government is more worried about the economic and social consequences of pollution. As a result, China's environmental issues are becoming worse due to escalating tensions between the country's need to protect the environment and its desire to grow economically.

China is progressively shifting from a focus on quick economic growth to a focus on high-quality economic development. In today's world, the global economy must undergo a green transition. Entrepreneurship in China's cities is greening because of a desire to use the environment to promote economic growth, according to recent research. Sustainable green growth is an inextricable aspect of sustainable development and a quality-development method that enables nations to overcome old technologies in a variety of areas through the utilization of energy-efficient and clean technology. For that aim, China has to take action to establish enabling conditions for the development of energy-efficient and clean technology, including laws and practices in its own nation and abroad, as well as technological transfer. Innovation in technology, environmental legislation, government involvement, industrial cooperation, utilization of renewable energy, and green total factor productivity are all covered in the context of “China's manufacturing and logistics business.”

Reducing pollution and the negative impact of heavy industry's dispersion on public perception are two critical components of economic reform's long-term success. Urban green infrastructure serves to emphasize the value of nature in urban settings. It has emerged in urban studies as a focus on the economics of financing urban green infrastructure programmes, such as park construction, urban stream restoration, and urban farm creation. Many of these programmes are aimed at attracting new economic investments and providing a green premium for real estate development by promoting a cleaner, greener image for communities, among other things. A natural, green trail built on protected linear corridors would enhance the environmental aspects and provide opportunities for outdoor recreation. With footpaths and/or cycle ways that are surrounded by trees, streams, and other natural features that frequently pass between urbanized areas and rural areas in China, this notion is realized.

Greenways have been reproduced around the country after receiving very good public reaction since their prototype development in 2010. However, greenway development is associated with some problems. A comprehensive survey on problems in greenway development and countermeasures for green economic development using Internet technologies is less investigated. As a result, this study analyses the issues and solutions related to China's greenway economic development from the perspective of the Internet and computers. The advantages of greenway in economic development and social well-being of Chinese people are also presented in this review. In addition, applications of smart computer Internet technologies in enhancing greenway planning and green economic development of China are provided in this paper.

## 2. Need for Greenway Development

A greenway is a kind of open, green area that runs the length of a city or town. Natural and manmade corridors like valleys, rivers, mountain ranges, and landscaped highways are common places for this kind of development to take root. Walking and cycling paths may be found throughout the park. Major parks and natural reserves are linked with historic sites and urban and rural communities. Because of their linear, connecting design, greenways are distinct from parks and other alternate open spaces observed in cities. A national programme may sensibly encompass green infrastructure and activities such as tree planting on highways, permeable vegetation on the surface, drainage basins, and green corridors inside these protected areas. To achieve sustainable development, it is necessary to properly harness natural resources as well as human resources, capital generation, and technology use [3]. The benefits of greenway development are explained in the following section and also depicted in Figure 2.

### 2.1. Tourism and Quality Economic Development

Greenways may be linked to tourism, serve as new tourist sites, and contribute to the economic growth of the areas they pass through. As a result, a tourism-related concept of greenways might offer the opportunity of generating new permanent tourist attractions, lowering seasonality in visitor flows, and establishing tourism brands. Increased growth of greenways in tourist destinations through the establishment of pathway networks provides more pleasant routes for travel by bicycle or on foot across the regions, allowing tourists to better understand the region's culture, heritage, and landscape. This will contribute to the region's overall economic development and decrease CO_2_ emissions. As a result, it is critical to make studies on whether investments in greenways deliver both economic and environmental benefits accessible to the political authorities and scientific community. One method of analyzing such economic data is to compare the costs of using greenways to the expenses of building infrastructure. Visitors come to Greenway from all over the world. It is not uncommon for towns to see the economic benefits of attracting visitors to these popular tourist attractions. Construction and maintenance jobs, as well as tourism-related possibilities such as river rafting trips, bicycle renting, restaurants, and hotels, are all encouraged by the development of trails and greenways.

Green infrastructure allows towns to be certified as protected tourism destinations. One billion visitors and one billion possibilities were coined by “the United Nations World Tourism Day Conference” in 2015 to emphasize the tourism industry's power to influence people's environmental behaviour. According to research, approximately 93% of Chinese tourists are choosing eco-friendly destinations when making vacation plans, and this trend is expected to continue in the future [4]. From a purely ecological perspective, Shanghai's ecological green belts have developed into both ecological and recreational spaces [5].

### 2.2. Psychological Well-Being

It is predicted that by 2050, more than 70 percent of the globe's population will live in cities, as per the “World Health Organization, 2013.” There are 78% of Taiwanese people living in urban areas, according to the “Directorate General for Budget, Accounting, and Statistics, 2018.” As urban green space disappears, so does the opportunity for urban people to interact with nature. With almost 20% of the population over the age of 65, Taiwan is on course to become a “super-aged” society by 2026 [6]. One-fifth to one-ninth of those 65 and older suffer from depression [7]. Suicide is more common among older people in Taiwan than in other age groups, and it climbs with age. Researchers, health care providers, and communities are now giving closer attention to older adults, which includes not only disease therapies but also effective psychological transitions, the advent of a healthy lifestyle, participation in physical activities, and societal engagement [8].

It is critical to maintain and prolong the lives of older persons, and urban green areas give senior inhabitants accessible access to nature. For example, UGWs are open spaces with varying widths that run parallel to roads and provide public access for recreational purposes. It is possible that greenways may improve the environment of urban regions, replace the lack of green space in advanced metropolitan regions, and offer stress-relieving and recreational possibilities for urban residents, strengthening their emotional links to the area [9]. There has been a lot of research on the advantages of urban green spaces, but most of it has concentrated on park visitors rather than those who live near them. People over the age of 65 in Taichung, Taiwan, prefer to spend time in parks close to their homes because of the importance of design, location, and upkeep.

Greenways may help communities improve their health by providing a safe, designated place for fitness activities, leisure, and walking and cycling (nonmotorized transportation) [10]. The health advantages of UGCs have been shown in several cross-sectional research studies. The causal link between UGC and inhabitants' physical and mental health, on the other hand, is yet unknown [11]. Using a natural experimental study approach, [12] investigated the influence of a large-scale UGW, the “102-kilometer-long East Lake Greenway in Wuhan, China,” on inhabitants' health outcomes. For elderly individuals to retain an active lifestyle, urban green areas are crucial. UGWs not only offers a physical environment that encourages older persons to get involved in outdoor activities in their communities, but they also provide social capital and social cohesiveness. As a result, the accessibility of these sites promotes older individuals' engagement in outdoor activities [13]. They facilitate social interaction and community cohesion by providing a natural gathering spot for locals.

### 2.3. Environmental Preservation

To minimize habitat fragmentation and manage the principles of natural ecosystems, UGCS are “multifunctional linear green spaces.” Greenways provide a wide range of benefits, including flood control, soil stabilization, water purification, and more. Green infrastructure refers to linked networks of green areas that may help with water quality enhancement, stormwater management, and wildlife conservation, among other things [14]. In China, the emphasis on greenway building is changing from production conservation and aesthetics to ecological protection [15]. In order to encourage new secondary sectors, such as production and innovative materials manufacture, the municipal government needs a clean environment. Maanshan's emergence as a tourist destination, real estate market, and other service sectors demands an appealing landscape and a good quality of life, which necessitates innovative approaches to mobilize and strengthen Maanshan's natural benefits in China. To date, Maanshan's environmental competitiveness has been bolstered by the municipal government's long-term focus on environmental protection. The presence of the ecological green belt is utilized to efficiently regulate urban land development and fulfill ecological operations such as “biodiversity maintenance, enhancement of overall protection and use of environmental resources in rural areas, regulation of the microclimate in cities and pollution absorption” [16]. Recently, academics have focused more on the compound operations of a green belt surrounding a city, and they've looked into new green belt planning strategies to assure the long-term growth of an ecologically protective green belt that can contribute to today's cities [17]. Green infrastructure may take the shape of multifunctional ecological networks that are natural, semi-natural, or manmade. New forms of transportation, entertainment, leisure, environmental preservation, cultural conservation, as well as protection against natural calamities like wind, soil erosion, and floods, have historically been connected with greenways.

### 2.4. Problems in China's Greenway Construction and Sustainable Economic Development

The greenway is associated with several benefits regarding economic, environmental, and individual aspects. But the implementation of an effective greenway in China is linked with certain challenges, which are explained below.

#### 2.4.1. Legal Issues

The rate of urbanization in China is increasing at a fast speed, but the building of UGCs has not kept pace with this rapid growth. As a primary factor, China lacks a legislative framework for UGCs, which is one of the main causes. Even while the People's Republic of China Urban and Rural Planning Law explicitly states that the green channel is an essential aspect of China's national greening, most of the relevant implementation depends on this law. As far as we know, there are no specific legislative requirements or indications that the UGC building is important for city planning and growth. In contrast, the relevance of UGC buildings has not been stressed in the design of urban infrastructure. To speed up the building of UGCs, a thorough legislative and regulatory framework is required.

#### 2.4.2. Lack of Environmental Awareness

China's economy rose at an annual rate of 9.7 percent after reform and opening up, propelling it to the position of the globe's second biggest economy [18]. Anyhow, China's heavy utilization of energy and the environment for economic expansion has resulted in a number of economic and social issues. Since China has become the world's top energy user, the World Bank has highlighted this fact. The reduction of CO_2_ emissions in China, which accounts for 26.6 percent of the globe's total emissions, is very difficult. In 2018, China was placed 120^th^ out of 180 nations in terms of environmental performance [19]. As of 2010, the price of environmental deterioration in China has climbed from 3% of GDP to 3.5% of GDP during the period from 2004 to 2010. To sum up, environmental deterioration in China is endangering the country's long-term growth. A lack of societal engagement in the greenway design might have a negative effect on the greenway's aims and priorities, notably its ecological functions [20, 21]. One of the most difficult aspects of greenway development is how to get local government agencies, community organisations, and other interested parties to participate in the planning and decision-making procedure. For the sake of environmental sustainability, it is critical to understand and change human behaviour.

To reduce the possible detrimental impact of technological growth on human and environmental health, it is required to properly address difficulties like rising energy usage, waste and greenhouse gas emissions, and the utilization of natural and nonrenewable raw resources. A greener future is one that replaces current technology, the Internet of Things (IoT), and the economy with environmentally friendly options, each of which has the potential to increase human well-being dramatically and so contribute to a more sustainable smart world [22].

#### 2.4.3. Planning and Management Issues

Landscape variety is an underappreciated contributor to a greenway's visual appeal and ecological diversity. When it comes to greenway alignment design, site appropriateness is the most important factor. The “one-size-fits-all” approach to greenway planning actions has resulted in the composition and variability of greenways in Shenzhen, making multifunctional greenway development in urban areas difficult [23]. UGCs' diverse landscapes will need greater attention in the future, as will the tactics for improving them in light of particular policy objectives.

China's cities are rapidly expanding and becoming denser. In turn, this puts more strain on the city's open spaces, hindering the growth of urban green infrastructure. Existing green spaces in highly populated areas have significant challenges, which raise questions about ensuring that all inhabitants have equitable access to urban green spaces. In order to enhance greenway planning in other cities, it is important to record and reflect on successful greenway design practices in emerging cities [24].

In an ideal world, roads would be as ecologically friendly as possible while also having aesthetically pleasing features to reduce the amount of environmental harm they cause. Researchers, engineers, and artists must collaborate to reshape human environments by designing roads depending on more than just engineering concerns; future roads must take ecological concerns into account but also have aesthetic properties to meet the needs for environmental protection during road construction [25]. Artistic landscapes can only be achieved via collaboration between science and artists [26]. Another important issue in greenway planning is the lack of innovative, energy-efficient technologies. A massive transportation network (railway, highway, and so on) has been created as a result of this rapid economic development and growth, including environmentally sensitive locations like Tibet that need careful engineering to protect the environment.

#### 2.4.4. Limited Concern on Visitor's Experience

Tourists' perceptions regarding greenways and eco-friendly locations are critical in developing an effective greenway development strategy. Previous greenway research has largely focused on physical-ecological design difficulties, with little concern for visitor experience [27]. Only a tiny number of greenway scholars have looked at visitors' personal values and established the degree to which such values are helpful in understanding tourists' motivation and making responsible judgments. Residents who reside near greenways have gotten minimal consideration in this design [28]. Though studies have looked at users' attitudes and preferences for greenways, little focus has been devoted to the changes in perceptions between nonresidential and residential users. Previous greenway research has viewed greenway users as single aspects, intercepting all greenway users, whether they are local residents, tourists, or people who go to the greenway from other regions of the city. While considering all greenway users and considering them as a single entity has offered important insights into the overall preferences of users and utilization patterns, it fails to distinguish between residential and nonresidential perceptions, resulting in broad management suggestions that may be in conflict with residential preferences [29]. Those who live near greenways are possibly the most significant stakeholders, as they must struggle wwith both the beneficial and negative consequences of greenways in their communities. Because local people have the most access to the greenway, which acts as a transportation and recreational corridor for their surrounding communities, their opinions, concerns, and preferences are possibly more significant than those of commuting users [30].

### 2.5. Countermeasures for Effective Greenway Economic Development

The technological innovations in the computer Internet provide better solutions for greenway development and sustainable economic development. Some of the countermeasures for effective greenway economic development are discussed below.

#### 2.5.1. Effective Policymaking

Many municipal development plans tend to recognize that environmental protection is quickly becoming a must for economic success rather than a choice. Despite the rising physical and political constraints imposed by the environment, China's governments have started to address environmental problems as part of their objectives to keep their cities' economies growing. Urban economic and environmental governance, according to this perspective, calls for a holistic approach rather than a fragmented one. In order to align their goals with those of the environmental movement, China's development regimes are becoming increasingly interested in implementing environmental laws in their cities.

After the Guangdong Provincial Government created the “Pearl River Delta (PDR) greenway network” in 2010, China's contemporary greenway movement was born. The PDR greenway network was designed to reduce gaps between urban and rural areas in terms of economic, environmental, and social factors [1]. Greenways have been more popular in China, with 31 provinces planning or implementing provincial greenways and 163 cities working on municipal greenways by the end of 2016. According to the “Ministry of Housing and Urban-Rural Development,” greenways have been officially acknowledged as a new national policy by the federal government.

Road development in China's Hubei Province's Shennongjia area since 2006 has seen a shift away from traditional methods, which were costly and harmful to the environment. This time, the goal is to build “aesthetic greenway systems” that safeguard both nature's ecosystem and society's values, resulting in environmentally and socially harmonious road networks. In China, this means that the networks account for Chinese aesthetic principles while also being in harmony with the environment and society's economic growth.

#### 2.5.2. Environmental Education Programs

To promote ecological consumerism and proenvironmental behaviour, environmental education is essential. We must never lose sight of our basic goal in environmental education: spreading environmental awareness to the general public. As a result of these arguments, environmental information and education have been included as two of the most important determinants of environmental knowledge [31].

The livelihoods of conservation participants across the globe have been radically transformed, and other socioeconomic processes have been impacted. In order to be successful, such conservation projects need to be well understood by the public. The Grain-for-green programme (GGP), the biggest conservation initiative in the world, has so far shown little proof of its impact on the lives of its members. Research by [32] examined whether the GGP programme achieves its purpose of protecting participants' lives while also improving their environmental awareness. Educational awareness programs, according to [33], consider the following aspects:

- Must enhance awareness regarding environmental conservation
- To facilitate personal reflection on environmental actions

(iii) Must support the application of environmentally sustainable behaviours

#### 2.5.3. Greenway Planning Using Computer Internet Technology

Tourists and the growth of service industries may be encouraged by efficient planning of greenways in rural areas.  Figure 3 shows the Internet technologies used in greenway planning and greenway approaches. It is possible to identify and demonstrate UGC planning techniques by analyzing the recent UGC structure and relating physical aspects to theories on “landscape architecture and ecology” as well as technologies like geographic information system (GIS), remote sensing, and graph theory [34].

The Shenzhen greenway network's activity distribution is mapped using a GIS. In their research, they have shown that greenways with dense housing, mixed land use, sophisticated street network, and huge parks enhance physical activity. An area's natural circumstances and level of environmental degradation must be taken into consideration before designing any greenway network. Afforestation requirements may be determined based on this information. A novel computer modeling technique, a tree belt modeling system (TBM), is proposed to assess the suitability of a particular location for greenway services [35]. TBM is a predesign step in the creation of an ideal greenway structure that determines whether or not tree belt functions will be available in the proposed network.

Using data fusion and computer virtual reality (VR), the work in [36] undertakes a study on urban green landscape design to illustrate the potential of a more planned design. SketchUp software is used to create models, and a digital camera is used to take continuous digital photos. To begin, a panoramic picture is created by stitching together many individual digital landscape photographs. For final tweaks to materials and lighting, they upload the reduced version into our VR platform, where they can compare it to the original model's volume and do a plan check. It is important to note that the study in [5] analyses greenway branding as a sort of green resource branding with a specific focus on “media promotion, users' outdoor activity trajectories, and the picture content of geotagged images.” Participation of outdoor users in greenway development may enhance their enjoyment of the greenway's benefits.

GIS was used in [37] in order to build a greenway. There were three different greenway alignment scenarios offered in [38], each based on the criteria of compatibility, variety, and integration in Wuchang, China. Incorporating land appropriateness and variety in the environment, they came up with the concept of a greenway potential index. Combining the greenway potential index and connectivity research, they found an ideal route for future greenways between their origin and destination that met both site suitability and landscape variety criteria. The study in [39] intended at determining the best way to build urban ecological landscapes using edge computing from the Internet of Things.

*(1) Green Comple*. In China, fast urban expansion has been reduced by the employment of several green-space planning techniques. For instance, Shanghai, Chengdu, and other megacities have created an ecological network of green spaces, while Beijing has established a greenbelt surrounding the city. However, because of the scarcity of available land and the low demand for natural space, encroachment and fast urban growth have persisted. Therefore, in the context of modern megacity growth, green space with a single purpose and single shape may not be the ideal option.

*(2) Green Ecological Corridor*. The green ecological corridor is a key component of the landscape's overall security and stability because it serves as a conduit for energy flows between various ecological source patches, a link between people and the environment, and a link between urban and rural regions. According to a review study, the role, connotation, denotation, and construction methods of the green ecological corridor have been significantly expanded and altered from the Emerald Necklace-style Park corridor system in the Boston area in the 1960s to the European Ecological Network in the early 21st century. The expansive Three-North Shelter Belt in dry areas is only one of several instances of green ecological corridors in China at various dimensions.

*(3) Greenway Network*. The most frequent human activity and the most powerful interference are connected to roads. Urbanization and an increase in vehicles have led to the creation of several broad major roadways in recent years. The road network's density has continuously risen, improving travel convenience and enhancing the connectivity between cities. However, forests and other natural environments have been fragmented as a result. The creation of a network of greenways, which connects roads with nearby greenery, can increase the amount of public space available for urban residents' leisure and recreational activities as well as the ecological areas available for wildlife to live and migrate. Greenways can also play a crucial role in a region's overall ecological security and the advancement of sustainability.

*(4) Blue-Green Ecological Network*. The river is a crucial component of the urban environment since it has flowing, linear, and natural elements. Rapid development has resulted in the artificialization of many natural rivers over the last several decades, as well as a significant loss of wetlands. Along with other problems, rivers have lost some of their natural characteristics and are no longer as effective at filtering water. This might be the root of Beijing's severe urban floods and Wuhan's severe waterlogging, among other major Chinese cities. The sustained growth of human settlements depends on river ecological restoration and watershed management. Restoring watersheds and urban-rural ecosystems may be accomplished by enhancing river connections and using watershed resources to create a blue-green ecosystem.

*(5) Green Ventilation Corridor*. Numerous case studies have been published on how green areas actively control the temperature via means like ventilation, cooling, and air purification. Green ventilation corridors may improve city ventilation, bring in fresh air, and reduce the heat island effect. There is a noticeable cooling and humidifying impact in the green ribbon area. Recent years have seen a boom in studies on the connection between urban climate (wind and temperature) and green space.

#### 2.5.4. Significance of Internet Technology in Green Economic Development

Technology use that does not damage, overexploit, or deplete natural resources, reduces energy consumption, produces completely reused or reclaimed products, and reduces waste and emissions during production and use are the main goals of “green, environmental, or clean technology” [40]. In other words, green technology is characterized by environmentally sustainable design, manufacture, use, and disposal with little or considerable environmental effect.  Figure 4 depicts the differences between conventional and green production industry.

Sustainability in economic development is a major issue, and this study examines how greening technology might help to improve the environment and economy while also enhancing human well-being and global modernity in the process [41]. According to research, Internet technologies have the potential to transform and bring numerous benefits (among them customer satisfaction, environmental protection, and increased profit) in a wide range of industries using the latest technology approaches and solutions, as well as eliminate or minimize the negative impact on human health and the environment. Information and computer technology (ICT) development has a favourable influence on boosting green total factor energy efficiency (GTFEE) and this role is controlled by environmental restrictions [42]. GTFEE is influenced by ICT development in various ways depending on the intensity of environmental control. In addition, the influence of ICT development on GTFEE varies greatly from area to area. It is possible that ICT infrastructure might play a big role in reducing carbon emissions from companies in the industrial sector. Industries may reduce their use of resources by using ICTs [43]. The study in [44] stated that the rise in ICT cuts carbon dioxide emissions in China.

## 3. Statistical Analysis

In statistical analysis, we use chi-square test and ANOVA test.

### 3.1. Chi-Square Test

The chi-square analysis is one of the most efficient statistical tools for testing a hypothesis when the factors are minimal. Unlike the other statistics, the chi-square may provide specific information on not just the importance of any significant variability but also which groups are responsible for those distinctions.

(1) $$\begin{array}{c} \sum y_{j-k}^{2}=\frac{{\left(P-F\right)}^{2}}{F}. \end{array}$$

Here, *P* = present point, *F* = real point, *Y*^2^= Chi-square value, and ∑ *Y*^2^ = To total all of the cell chi-square values, whether they had been treated or not, the following formula is used to calculate expected chi-square values:

(2) $$\begin{array}{c} F=\frac{N_{S}\times N_{D}}{o}, \end{array}$$

where *F* = reflects the work value of the unit, *N*_*D*_ = denotes that cell nucleus row edge, *N*_*S*_  = denotes that cell's row edge, and *o* = reflects the sample group as a whole.

The sample size is split by the product of the row marginal and the column marginal for each cell.

(3) $$\begin{array}{c} y^{2}=\frac{{\left(P-F\right)}^{2}}{F}. \end{array}$$

Correlation measures are statistical assessments of the strength of a relationship. The Cramer's *V* test is the most often utilized chi-square strength test. Using the formula, it is easy to calculate

(4) $$\begin{array}{c} \sqrt{\frac{y^{2}/o}{\left(l-1\right)}=\sqrt{\frac{y^{2}}{o\left(l-1\right)}.}} \end{array}$$

The chi-square is a useful data analysis tool that reveals a lot about the nature of research data.

### 3.2. ANOVA

Analysis of variance, or ANOVA, is a quantitative tool for dividing reported variability data into multiple parts for use in subsequent tests. A one-way ANOVA has been used to discover the relationship between variables when there are 3 or more data sets. The classic ANOVA F-statistic is the proportion of average sums squared of the null model with an anthropic principle to the whole model. The parameters are calculated using the least-squares approach, with all variances being identical. This may be expressed as

(5) $$\begin{array}{c} S=\frac{MH_{\text{between}}}{MH_{\text{error}}}, \end{array}$$

where

(6) $$\begin{array}{c} MH_{\text{between}}=\frac{\sum_{i=1}^{k}l{\left(\bar{x}-\bar{x}\right)}^{2}}{n-1}. \end{array}$$

Also,

(7) $$\begin{array}{c} MH_{\text{error}}=\frac{\sum_{i=1}^{k}\sum_{j=1}^{l_{i}}{\left(x_{ij}-x_{i}\right)}^{2}}{l-k}. \end{array}$$

The Welch-test-statistic is defined as

(8) $$\begin{array}{c} Y=\frac{\sum_{i=1}^{K}y_{j}\left[{\left(x_{i}-\tilde{x}\right)}^{2}/\left(K-1\right)\right]}{1+2\left(K-2\right)/K^{2}-1\sum_{i=1}^{K}\left[{\left(1-y_{j}/u\right)}^{2}/\left(l_{i}-1\right)\right]}, \end{array}$$

where *l*_*i*_ =  *n*/*t*_1_^2^, *u* =  ∑_*i*=1_^*K*^*l*_*i*_, and *Y*=1/*u*∑_*i*=1_^*K*^*l*_*i*_*y*_*j*_; we have

(9) $$\begin{array}{c} S=\frac{k^{2}-1}{s\sum_{i=1}^{K}\left[{\left(1-y_{j}/u\right)}^{2}/\left(l_{i}-1\right)\right]}. \end{array}$$

The Brown–Forsythe-test-statistic is defined as

(10) $$\begin{array}{c} S^{*}=\frac{{\sum_{i=1}^{K}o\left({\bar{x}}_{j}-\bar{x}\right)}^{2}}{\sum_{i=1}^{K}\left(1-l_{i}/H_{i}^{2}\right)}. \end{array}$$

When *L*_*o*_ is factual, the allocation of *S*^*∗*^ is appropriate by a central *S* distribution with degrees of freedom *K* − 1 and *s*, where *s* is defined as

(11) $$\begin{array}{c} \frac{1}{s}=\frac{\sum_{i=1}^{K}c_{i}^{2}}{\left(l_{i}-1\right)},\;c_{i}=\frac{\left(1-l_{i}/H_{i}^{2}\right)}{\sum_{j=1}^{h}\left(1-l_{i}/H_{i}^{2}\right)}. \end{array}$$

To calculate the generalized *p* value, the generalized *p* value is now computed as *p* = 1 − *r*, where *s* is the sample size.

(12) $$\begin{array}{c} s=A\left(J_{k-1l-k}\left(\frac{l-k}{k-1}{\tilde{t}}_{b}\left(\frac{l_{1}t_{1}^{2}}{B_{1}B_{2},\ldots ,B_{K-1}},\frac{l_{2}t_{2}^{2}}{B_{1}B_{2},\ldots ,B_{K-1}},\frac{l_{3}t_{3}^{2}}{\left(1-B_{2}\right)B_{3},\ldots ,B_{K-1}},\ldots \frac{l_{1}t_{K}^{2}}{\left(1-B_{K-1}\right)}\right)\right)\right). \end{array}$$

The prediction is calculated with regard to separate Beta stochastic process in an *F*-distribution having *h* − I, *V* − *h* dof.

(13) $$\begin{array}{c} B_{K}∼\text{Beta}\left(\sum_{i=1}^{k}\frac{\left(l_{i}-1\right)}{2},\frac{\left(l_{k+1}-1\right)}{2}\right),\;l=1,2,\ldots ,k-1. \end{array}$$

The *p* value is calculated by numerically integrating the anticipated value in the *p* value formula with regard to the Beta random variables.

## 4. Conclusion

China's recent growth has been the quickest among the world's major economies. Many nations have been able to change from a development mode focused only on economic expansion to one that prioritizes resource conservation and environmental preservation via green economic growth. An urban green area provides a secure and healthy atmosphere that is ideal for physical and recreational activities as well as for social contact. This paper presents a comprehensive review of problems and solutions for greenway economic development in China. The survey clearly emphasized the advantages of greenways for socioeconomic, individual, and environmental development. In addition, the challenges in greenway development like legal, planning, and environmental awareness issues are explained in detail. Finally, the importance of Internet technologies in greenway planning and green economic development is illustrated. Hence, this survey provides detailed insights into greenway development for greenway researchers and designers.

### 4.1. Future Work and Recommendation

The findings point to ramifications for the future design and development of greenways, with a particular emphasis on safeguarding the rights of private landowners in addition to the public's right to a healthy environment. Directions for future study should centre on investigating the ways in which information-education initiatives have the potential to greatly raise community awareness and understanding of the advantages of greenway corridors. The findings of the study point to the need to do more research into a number of topics, each of which has the potential to provide vital information that will be relevant to the future design and development of rural greenways. It is recommended that a continuing and in-depth investigation and analysis of the differences in people's perceptions of streamland be carried out, with the comparison being made between rural homeowners of agricultural land, rural homeowners of nonagricultural land, suburban homeowners, and urban residents. Pursuing research that aims to lead to the creation of information-education programmes that prioritise environmental quality, aesthetics, and cultural-historical preservation should be a priority. These programmes should enhance community and landowner understanding of the advantages that streamlands provide.

## Figures and Tables

**Figure 1:** Relationship between environmental degradation and economic development.

**Figure 2:** Overall advantages of greenways.

**Figure 3:** Computer Technology in greenway approaches.

**Figure 4:** Green economic development.

## Data Availability

The data used to support the findings of this study are available from the author upon request.
